The article "A Study on the Effect of Nursing Intervention Based on Health Behavior Change Integration Theory on Patients with Limb Fracture and Its Effect on Limb Function and Self-Efficacy" was retracted in 2023. Reasons: signs of a paper mill; suspected computer-generated content; unreliable results or conclusions; lack of ethics approval or compliance.

# A Study on the Effect of Nursing Intervention Based on Health Behavior Change Integration Theory on Patients with Limb Fracture and Its Effect on Limb Function and Self-Efficacy

**DOI:** 10.1155/2022/1621210

**Published:** 2022-07-13

**Authors:** Shunhong Luo, Yu Xie, Shangwen He, Jian Li, Chunhua He

**Affiliations:** ^1^Department of Joint and Hand Surgery, The First People's Hospital of Huaihua (Jishou University of the Fourth Affiliated Hospital), Huaihua, Hunan, China 418000; ^2^Operation Room, The First People's Hospital of Huaihua (Jishou University of the Fourth Affiliated Hospital), Huaihua, Hunan, China 418000

## Abstract

**Objective:**

To assess the impact on nursing care based on the theory of health behavior change integration in patients with limb fracture and its effect on limb function and self-efficacy.

**Methods:**

The starting and ending time of this study is from February 2021 to February 2022. In this study, 116 hospitalized patients with limb fracture were selected as the object of study. According to the method of random number table, the patients were divided into study group and control group. The patients of the study cohort were given nursing healthcare based on the theory of health behavior change integration, while those in the control cohort were given common nursing. The scores of self-rating anxiety scale (SAS), self-rating depression scale (SDS), Frankl compliance scale, self-efficacy scale (GSES), activity of daily living scale (ADL), and Fugl-Meyer limb motor function assessment (FMA) were studied before and 3 months after nursing.

**Results:**

After 3 months of nursing, the SAS and SDS scores of the study group were lower than those of the control group, and the difference between groups was statistically significant (*p* < 0.05). After 3 months of nursing, the scores of Frankl scale, GSES, ADL scale, and FMA scale in the study group were higher than those in the control group, and the difference between groups was statistically significant (*p* < 0.05).

**Conclusion:**

The value of nursing interventions based on the integration of health behavior change theory is even more significant in patients with limb fractures. It is more helpful in reducing patients' anxiety and depression, increasing compliance and improving limb function. Self-efficacy and daily living skills were also significantly improved.

## 1. Introduction

Limb fracture is a common disease in clinic, accounting for more than 70% in orthopaedics. This disorder is more common in patients with external stress or osteoporosis [1]. The patients with limb fracture will have varying degrees of swelling and pain, and joint function exercise and incision healing will be seriously affected after operation, which can cause adverse reactions such as fracture healing and prolonged rehabilitation time of joint activity function [2]. With the rapid development of transportation and construction industry, more and more patients have broken bones due to traffic accidents or falling from height [3]. Meanwhile, because of comminuted fracture, poor reduction, weight-bearing, infection, and other reasons, some patients still have nonunion fracture, which seriously affects the prognosis and quality of life of patients, increasing their physical pain and economic burden [4]. The patients with limb fracture will experience varying degrees of swelling and pain, which seriously affect joint function training and postoperative incision healing, resulting in fracture healing and joint range of motion recovery time prolonged [5]. Therefore, it has become a major clinical problem to seek a treatment with good therapeutic effect and fewer side effects [6]. Fractures are usually treated by surgery, and postoperative fractures and surgical trauma are accompanied by varying degrees of pain and swelling [7]. It is necessary to implement early functional exercise combined with positive and effective nursing intervention measures to improve patients' self-management ability, effectively improve the postoperative rehabilitation quality of patients' joints, and promote the recovery of limb function.

The article "A Study on the Effect of Nursing Intervention Based on Health Behavior Change Integration Theory on Patients with Limb Fracture and Its Effect on Limb Function and Self-Efficacy" was retracted in 2023. Reasons: signs of a paper mill; suspected computer-generated content; unreliable results or conclusions; lack of ethics approval or compliance.

The occurrence and development of four-limb fracture are closely related to the bad behavior habits of patients. Because patients are often at home, medical staff cannot always become supervisors and guides of their behavior changes. The patients need to learn and persevere in self-management, so helping patients to form good self-management behavior is one of the main goals for nurses to implement health intervention and behavior intervention [8, 9]. Among them, the term “self-management (selfmanagement)” was first put forward by Creer in the study of childhood asthma [10]. However, most of the existing studies adopt the definition of Lorig and Halsted [11, 12]. “Self-management” means that patients improve and maintain their own health through personal behavior, manage and monitor the symptoms and precursors of their own disease, and reduce the impact of disease on personal social function, interpersonal relationship, and emotional function. Long-term outcomes adhere to the management of their own diseases of a healthy behavior. Previous studies at home and abroad have shown that through self-management, patients can give full play to their subjective initiative, promote the change of bad behavior, and acquire the ability to actively deal with and solve health problems, thus changing the quality of life [13]. In another study, after implementing diversified health education intervention for 3 months, the self-efficacy and quality of life of patients were significantly enhanced [14].

The article "A Study on the Effect of Nursing Intervention Based on Health Behavior Change Integration Theory on Patients with Limb Fracture and Its Effect on Limb Function and Self-Efficacy" was retracted in 2023. Reasons: signs of a paper mill; suspected computer-generated content; unreliable results or conclusions; lack of ethics approval or compliance.

In order to effectively improve patients' self-management skills, we need to start not only by imparting knowledge and information to patients but also by combining it with behavioral interventions [15–17]. In previous studies, although the theory of health behavior change has changed the behavior of patients, it cannot be maintained for a long time. The self-efficacy theory can improve the confidence of patients; however, it ignores the social and physical effects of patients. Social promotion theory emphasizes the influence of environment on patients but ignores the influence of patients' psychological and physical function. Although there were many theories in the past, they often only focused on the unilateral of the patient. American nursing expert Ryan proposed a dynamic and integrated patient-centered theoretical model, the Integrative Theory of Health Behavior Change, in 2009, through interventions and theories related to health behavior change [18]. The theory emphasizes that the change of behavior is to enhance the ability of self-management and social support by learning knowledge and cultivating beliefs. In recent years, nursing intervention based on health behavior change integration theory is widely used in medical care. However, there are few nursing intervention studies based on health behavior change integration theory for patients with limb fractures in China. Therefore, this study selected 116 patients with limb fracture treated in our hospital from February 2021 to February 2022 as the research object to study the effect of nursing intervention based on the theory of health behavior change integration in patients with limb.

## 2. Materials and Methods

### 2.1. General Information

The starting and ending time of this study is from February 2021 to February 2022. In this study, 116 hospitalized patients with limb fracture were selected as the object of study. According to the method of random number table, the patients were divided into study group (*n* = 58) and control group (*n* = 58). The study group included 30 male patients and 28 female patients, whose age ranged from 48 to 65 years old (58.48 ± 3.27 years old). In the control group, there were 28 male patients and 30 female patients, whose age was from 47 to 66 years old (58.51 ± 3.31 years old).

Inclusion criteria are as follows: (1) the patients were in accordance with the Diagnostic Classification and functional Evaluation Standard of Bone and related injuries and Diseases; (2) there were no serious diseases in heart, brain, liver, kidney, and other important organs, no local skin infection, allergy, damage, and no serious diseases of blood system; and (3) patients voluntarily participate in the trial and sign the informed consent form.

The article "A Study on the Effect of Nursing Intervention Based on Health Behavior Change Integration Theory on Patients with Limb Fracture and Its Effect on Limb Function and Self-Efficacy" was retracted in 2023. Reasons: signs of a paper mill; suspected computer-generated content; unreliable results or conclusions; lack of ethics approval or compliance.

Exclusion criteria are as follows: (1) those who did not meet the diagnostic criteria and inclusion criteria; (2) pregnant women; (3) the cases were experiencing a history of mental illness; (4) those who could not adhere to treatment and had serious adverse reactions and failed to complete the observation course prescribed in the study; and (5) there were anti-infective and hormone therapy within 3 months before treatment.

### 2.2. Methods

#### 2.2.1. Technical Route

Technical route is shown in Figure 1.

#### 2.2.2. Intervention Scheme

The control group was accepted the routine nursing. (1) Preoperative nursing includes admission education and preoperative preparation and guidance. (2) Postoperative nursing includes close observation of the changes of postoperative vital signs, evaluation of patients' neurological function (including muscle strength, sensation, and excretion function), guidance of postoperative daily life (postural posture, dietary adjustment, hygiene maintenance, and excretion skills), teaching patients postoperative pain relief skills, guiding patients to correct functional exercise, prevention and management of complications, psychological nursing, and routine health education. (3) Discharge health guidance includes rehabilitation exercise, diet adjustment, fall prevention, medication, and other matters needing attention.

The study group was implemented nursing intervention based on the integration theory of health behavior change: (1) preoperative nursing including admission education and preoperative preparation and guidance and (2) 2-3 days after operation: (1) personalized assessment: based on routine assessment and baseline assessment, dynamic interviews were used to evaluate the disease cognition of patients with limb fractures and to guide patients to judge their own bad lifestyle and disease-related risk factors. Encourage them to talk about the harm of these bad living habits and risk factors to their health, and make them actively have the motivation to change their bad habits; (2) to guide patients to consider the possible benefits of changing bad health behavior and preventing controllable risk factors leading to brittle fractures, arouse patients' psychology of urgent change and arouse their motivation for active behavior change; (3) provide personalized disease-related health information for patients according to the above evaluation results, and teach patients how to apply it to life. Correct the misunderstandings of disease knowledge of patients and their spouses or caregivers, and provide correct knowledge guidance, including an overview of brittle fractures, prevention of refractures, improve their cognitive level of the disease, and make them have a sense of identity. Ask them to browse the manual repeatedly to stimulate patients' “health threat awareness,” to help patients establish a belief in promoting health; (4) patients are encouraged to report their willingness to change their behavior. The willingness scale (0-10 minutes 0 for “no behavior motivation” and 10 for “strong motivation”) was used to judge whether the patient was motivated for behavior change, and the patient chose the scale value according to his own condition. Studies have shown that patients with a score of more than 7 represent the transition from the behavioral intention period to the behavioral preparation period and are most likely to begin to take the behavior [19]. The next stage of intervention should be carried out for the volunteers with behavior change, and the unwilling volunteers should find out the cause and solve the problem; (3) 5-10 days after operation. Through motivational interviewing, patients are led to talk actively about the behavioral habits and goals that need to be changed. Changes can be made to achieve the goals and ways to self-monitor and self-evaluate. Evaluate the motivation of the patient's behavior change, and compared with the last score, those who have progress to the next step of intervention, if there is no willingness to change, it is necessary to find out the reason and deal with it in time; (4) 1-2 days before discharge. With the cooperation of doctors, nurses, patients, and their families, a patient's behavior change goal can be achieved one month after discharge, and the specific implementation plan is determined according to the actual situation of the patient. The patients are taught specific ways to manage relevant behaviors and are guided to train skills to manage adverse emotions and reduce stress during behavior change. The patients are encouraged to take the initiative to evaluate the effect and feedback the results to the medical staff in a timely manner. Once again, evaluate the motivation of the patients' behavior change, and summarize the contents of in-hospital intervention for those with higher scores. If the motivation score is below 7, the nurse should guide the patient to state the problems and doubts and give advice; (5) the patient was discharged from hospital for 1 month and 3 months. Within 1 month after discharge, push disease-related knowledge to patients through WeChat on time every week, remind patients to send self-management diary pictures, for poor compliance patients, phone follow-up or WeChat video communication, ask the reason, and deal with it. One month after discharge, the propaganda content was pushed every 2 weeks. The patients sent self-management diary chart, telephone, or WeChat video every week to follow up the patients and learned about the implementation of the patient's action plan through motivation interviews.

The article "A Study on the Effect of Nursing Intervention Based on Health Behavior Change Integration Theory on Patients with Limb Fracture and Its Effect on Limb Function and Self-Efficacy" was retracted in 2023. Reasons: signs of a paper mill; suspected computer-generated content; unreliable results or conclusions; lack of ethics approval or compliance.

### 2.3. Observation Index

1. The scores of self-rating anxiety scale (SAS) and self-rating depression scale (SDS) in the two groups were studied before nursing and 3 months after nursing. SAS ≥ 50 as anxiety, 50 ≤ SAS < 60 as mild to mild anxiety, 60 ≤ SAS < 70 as moderate anxiety, and SAS ≥ 70 as severe anxiety [20]. With the increase of the score, the degree of anxiety is more serious. The SDS takes the score > 52 as the standard to judge the depression state of the patients [21]. The standard score ≥ 53 is depression, 53-62 is mild depression, 63-72 is moderate depression, and more than 72 is severe depression. The higher the score, the more serious the depression
2. To study the scores of Frankl compliance scale before nursing and 3 months after nursing between the two groups. The highest score of Frankl is 4. The higher the score, the better the compliance [22]
3. To study the self-efficacy scale (GSES) scores of the two groups before nursing and after 3 months of nursing. The score of GSES ranges from 10 to 40. The higher the score, the higher the level of self-efficacy [23]
4. To study the activity of daily living scale (ADL) scores of the two groups before nursing and after 3 months of nursing. The highest score of ADL is 100. The higher the score, the stronger the ability of daily life [24]
5. To study the Fugl-Meyer limb motor function assessment (FMA) scores of the two groups before nursing and 3 months after nursing. The total score of FMA is 66. The higher the total score, the better the motor function [25]

### 2.4. Statistical Analysis

The statistical analysis of the data in this study used the SPSS24.0 software. The statistical graphics were drawn by GraphpadPrism8.0. The measurement data with normal distribution were expressed by mean ± standard deviation ($\bar{x}\pm s$). Paired sample *t*-test was used for intragroup comparison, and independent sample *t*-test was used for intergroup comparison. *p* < 0.05 was statistically significant. If it was not consistent, it was expressed by the median (lower quartile to upper quartile). Paired sample nonparametric test was used for intragroup comparison, and independent sample nonparametric test was used for intergroup comparison. The grade data were tested by FISHER accurate method, *p* < 0.05 indicated statistical significance.

The article "A Study on the Effect of Nursing Intervention Based on Health Behavior Change Integration Theory on Patients with Limb Fracture and Its Effect on Limb Function and Self-Efficacy" was retracted in 2023. Reasons: signs of a paper mill; suspected computer-generated content; unreliable results or conclusions; lack of ethics approval or compliance.

## 3. Results

### 3.1. The Scores of SAS and SDS before Nursing and 3 Months after Nursing in Two Groups

Before nursing, there was no significant difference in SAS and SDS scores between the two groups, and the difference between groups was statistically significant (*p* < 0.05). After 3 months of nursing, the SAS and SDS scores of the study group were lower than those of the control group, and the difference was statistically significant, and the difference between groups was statistically significant (*p* < 0.05). All the results are shown in Tables 1 and 2.

### 3.2. The Score of the Frankl Scale before and 3 Months after Nursing

Before nursing, there was no significant difference in the scores of the Frankl scale between the two groups (*p* > 0.05). After 3 months of nursing, the score of the Frankl scale in the study group was higher than that in the control group, the difference was statistically significant, and the difference between groups was statistically significant (*p* < 0.05). All the results are shown in Table 3.

### 3.3. The Scores of GSES before Nursing and 3 Months after Nursing in Two Groups

Before nursing, there was no significant difference in the GSES scores between the two groups (*p* > 0.05). After 3 months of nursing, the GSES score of the study group was statistically higher than that of the control group, and the difference between groups was statistically significant (*p* < 0.05). All the results are shown in Table 4.

### 3.4. The Scores of ADL Scale before Nursing and 3 Months after Nursing in Two Groups

Before nursing, there was no significant difference in the ADL scale scores between the two groups (*p* > 0.05). After 3 months of nursing, the ADL scale score of the study group was higher than that of the control group, the difference was statistically significant, and the difference between groups was statistically significant (*p* < 0.05). All the results are shown in Table 5.

### 3.5. The Score of FMA Scale before and 3 Months after Nursing

Before nursing, there was no significant difference in FMA scale between the two groups (*p* > 0.05). After 3 months of nursing, the score of FMA scale in the study group was higher than that in the control group, the difference was statistically significant, and the difference between groups was statistically significant (*p* < 0.05). All the results are shown in Table 6.

## 4. Discussion

With the rapid development of transportation and construction industry, there are more and more patients with fractures caused by car accidents [26]. The patients with limb fracture will have varying degrees of swelling and pain, and joint function exercise and incision healing will be seriously affected after operation, which can cause adverse reactions such as fracture healing and prolonged rehabilitation time of joint activity function [27].

The article "A Study on the Effect of Nursing Intervention Based on Health Behavior Change Integration Theory on Patients with Limb Fracture and Its Effect on Limb Function and Self-Efficacy" was retracted in 2023. Reasons: signs of a paper mill; suspected computer-generated content; unreliable results or conclusions; lack of ethics approval or compliance.

At present, surgical treatment of limb fractures can effectively alleviate the clinical symptoms of patients, but this only solves the disease problem of the fracture site and cannot fundamentally prevent the recurrence of fractures [28, 29]. The postoperative nursing intervention for patients with limb fracture is mainly to change their concept, adjust diet, strengthen functional exercise, and guide the correct use of drugs. However, the most middle-aged and elderly patients with memory loss have weak knowledge of disease prevention and nursing. In the lack of family and social support and supervision, the patients are difficult to adhere to postoperative rehabilitation-related treatment and functional rehabilitation exercise. The compliance of patients gradually decreased, seriously affecting postoperative rehabilitation. In turn, it increases the risk of postoperative complications and refracture [29]. Therefore, how to guide and improve the self-management ability of patients with limb fracture is an urgent problem for nurses to pay attention to and solve.

Some studies have shown that the maintenance of medical compliance is positively correlated with the level of patients' self-efficacy [30]. A high level of self-efficacy (individual confidence or belief in behavior change) has a positive impact on patients' behavior change, and patients will be willing to make active efforts and solve the difficulties encountered. The nursing intervention model based on the integration theory of health behavior change can enable doctors and nurses to better understand the process of behavior change and their effectiveness in guiding patients' behavior change. In order to provide patients with more standardized and detailed guidance and help patients establish and maintain healthy behavior, this nursing model has been widely used at home and abroad. The integrated theoretical framework of health behavior change consists of three models and two-phase results [31]. The three models are self-management model, knowledge and belief model, and social promotion model, in which self-management model is the core of health behavior change integration theory, and knowledge belief model and social promotion model are the basis of health behavior change integration theory. The integration theory of health behavior change emphasizes that only by improving patients' disease awareness, enhancing self-management skills, and creating a supportive environment can we promote the establishment and maintenance of patients' health behavior [32].

The article "A Study on the Effect of Nursing Intervention Based on Health Behavior Change Integration Theory on Patients with Limb Fracture and Its Effect on Limb Function and Self-Efficacy" was retracted in 2023. Reasons: signs of a paper mill; suspected computer-generated content; unreliable results or conclusions; lack of ethics approval or compliance.

The two stages of outcomes refer to short-term outcomes and long-term outcomes. The former refers to the initial establishment of behavioral change and the adoption of healthy behaviors, which can be achieved in a short period of time. The latter refers to the need for the patient to maintain healthy behaviors over time, moving from quantitative to qualitative change and reaching the long-term goal of improved health.

The patients will have an immediate sense of accomplishment after achieving their short-term goals. This sense of accomplishment will stimulate the patient's intrinsic motivation to carry out the next goal and avoid the problems that behavior changes are difficult to implement due to the utopian expectations of long-term goals. ITHBC is also widely used in the self-management of chronic diseases such as COPD patients, stroke, and atrial fibrillation surgery in China [33, 34]. It is indicated that it has good guiding significance for chronic disease self-management and bad behavior changes. Therefore, this paper carried out a study to study the effect of nursing intervention based on the integration theory of health behavior change in patients with limb fractures and its influence value on limb function and self-efficacy.

The results of the study showed that after implementing the nursing intervention based on the integrated theory of health behavior change, the scores of the SAS and SDS of the patients were lower than those of routine nursing (*p* < 0.05). The scores of the Frankl scale, GSES, ADL scale, and FMA scale were higher than those of routine nursing (*p* < 0.05). It is proved that the application value of nursing intervention based on health behavior change integration theory in patients with limb fracture is more significant. This is mainly because the integration theory of health behavior change guides the attention of behavior intervention. (1) Evaluation will run through the whole process of behavioral intervention, including individualized assessment of patients' perception of disease, individual-related disease risk factors, self-efficacy, and health beliefs, analyze the factors that affect patients' behavior for change, and judge the stage of patients' self-management behavior. (2) Family members or close friends are encouraged to join the patient in health management, to monitor and encourage each other, to reduce anxiety and depression, and to improve medical compliance. The patients with similar diseases can also be gathered by establishing WeChat groups to create a social support environment for patients. Teach patients to obtain continuous information support, emotional support, and evaluation support through the Internet, television, and other mass media, better maintain healthy behavior, actively cooperate with rehabilitation training, and promote the rehabilitation of limb function, improving the ability of daily life [35]. (3) Based on the results of the evaluation, patients are provided with individual knowledge of the disease, enhanced individual self-efficacy, and the building of health beliefs. Caregivers should work with patients to develop behavior change goals and implementation plans and instruct patients on how to change and accomplish them in their daily lives. Patients record health behavior change being recorded and being self-evaluated, reflecting the results to medical staff in real time. There are some limitations in this study. First, the sample size of this study is not large, and it is a single-center study, so bias is inevitable. In future research, we will carry out multicenter, large-sample prospective studies, or more valuable conclusions can be drawn.

The article "A Study on the Effect of Nursing Intervention Based on Health Behavior Change Integration Theory on Patients with Limb Fracture and Its Effect on Limb Function and Self-Efficacy" was retracted in 2023. Reasons: signs of a paper mill; suspected computer-generated content; unreliable results or conclusions; lack of ethics approval or compliance.

In conclusion, the value of nursing interventions based on the integration of health behavior change theory is even more significant in patients with limb fractures. It is more helpful in reducing patients' anxiety and depression, increasing compliance, and improving limb function. Self-efficacy and daily living skills were also significantly improved.

## Figures and Tables

**Figure 1:** Technology roadmap.

**Table 1:** The scores of SAS before nursing and 3 months after nursing in two groups.

Grouping	Before nursing (score)	After 3 months of nursing (score)	*t* value	*p* value
Control group (*n* = 58)	65.39 ± 4.17	50.15 ± 3.27	21.902	<0.01
Research group (*n* = 58)	65.42 ± 4.28	45.19 ± 2.04	32.495	<0.01
*t* value	0.038	9.801		
*p* value	0.969	<0.01		

**Table 2:** The score of SAS before nursing and 3 months after nursing in two groups.

Grouping	Before nursing (score)	After 3 months of nursing (score)	*t* *value*	*p* *value*
Control group (*n* = 58)	68.47 ± 5.44	51.46 ± 3.27	20.409	<0.01
Research group (*n* = 28)	68.53 ± 5.37	44.22 ± 2.17	31.965	<0.01
*t* value	0.059	14.049		
*p* value	0.952	<0.01		

**Table 3:** The score of the Frankl scale before nursing and 3 months after nursing.

Grouping	Before nursing (score)	After 3 months of nursing (score)	*t* value	*p* value
Control group (*n* = 58)	1.25 ± 0.19	2.68 ± 0.24	35.578	<0.01
Research group (*n* = 58)	1.28 ± 0.17	3.75 ± 0.04	107.711	<0.01
*t* value	0.896	33.492		
*p* value	0.372	<0.01		

**Table 4:** The GSES score of two groups before nursing and 3 months after nursing.

Grouping	Before nursing (score)	After 3 months of nursing (score)	*t* value	*p* value
Control group (*n* = 58)	19.12 ± 1.39	29.29 ± 2.15	30.253	<0.01
Research group (*n* = 58)	19.14 ± 1.27	35.25 ± 3.14	36.223	<0.01
*t* value	0.081	11.927		
*p* value	0.935	<0.01		

The article "A Study on the Effect of Nursing Intervention Based on Health Behavior Change Integration Theory on Patients with Limb Fracture and Its Effect on Limb Function and Self-Efficacy" was retracted in 2023. Reasons: signs of a paper mill; suspected computer-generated content; unreliable results or conclusions; lack of ethics approval or compliance.

**Table 5:** The score of ADL scale before nursing and 3 months after nursing.

Grouping	Before nursing (score)	After 3 months of nursing (score)	*t* value	*p* value
Control group (*n* = 58)	45.59 ± 3.06	76.18 ± 4.11	45.465	<0.01
Research group (*n* = 58)	45.63 ± 3.13	82.53 ± 5.24	46.042	<0.01
*t* value	0.069	7.262		
*p* value	0.945	<0.01		

**Table 6:** The score of FMA scale before nursing and 3 months after nursing.

Grouping	Before nursing (score)	After 3 months of nursing (score)	*t* value	*p* value
Control group (*n* = 58)	31.38 ± 2.19	50.59 ± 3.32	36.784	<0.01
Research group (*n* = 58)	31.42 ± 2.17	58.36 ± 4.14	43.894	<0.01
*t* value	0.099	11.150		
*p* value	0.922	<0.01		

## Data Availability

The datasets used and analyzed during the current study are available from the corresponding author upon reasonable request.

## References

[1] Liguang Y. (2017). Observation on the curative effect of traditional Chinese medicine fumigation therapy on 139 cases of fracture rehabilitation. *Henan Traditional Chinese Medicine*.

[2] Wang X. L., Zhu X. P., Ji D. X. (2018). Beneficial effect of traditional Chinese medicine fumigation "Bone-healing Powder" in postoperative pain and recovery of neurological function of traumatic thoracolumbar spine fractures: a case-control study. *Medicine (Baltimore)*.

[3] Feng Y., Hao B. (2021). Effect of nursing intervention on rehabilitation of patients with limb swelling after operation of limb fracture. *Minerva Medica*.

[4] Deli X., Hao L. (2015). Clinical study on the treatment of limb fractures with combination of traditional Chinese and Western medicine. *Journal of Traditional Chinese Medicine*.

[5] Ping L., Xingping D. (2018). Curative effect observation and nursing of traditional Chinese medicine fumigation after operation of supracondylar fracture of humerus. *Chinese and Foreign Health Abstracts*.

[6] Galing H., Weihong M. (2017). Application of traditional Chinese medicine fumigation in the rehabilitation of traumatic fractures of extremities. *The Psychiatrist*.

[7] Jihong D., Li J. (2018). Application of traditional Chinese medicine fumigation in rehabilitation nursing after fracture operation. *Nursing Practice and Research*.

[8] Inagawa T., Hamagishi T., Takaso Y. (2013). Decreased activity of daily living produced by the combination of Alzheimer's disease and lower limb fracture in elderly requiring nursing care. *Environmental health and preventive medicine*.

The article "A Study on the Effect of Nursing Intervention Based on Health Behavior Change Integration Theory on Patients with Limb Fracture and Its Effect on Limb Function and Self-Efficacy" was retracted in 2023. Reasons: signs of a paper mill; suspected computer-generated content; unreliable results or conclusions; lack of ethics approval or compliance.

[9] Liu H., Wang Y., Li M., Chen D., Tang Y. (2022). Compliance of functional exercises in school-age children with limb fractures: implication for nursing countermeasures. *BMC pediatrics*.

[10] Lorig K. R., Halsted H. (2003). Self-management education: history, definition, outcomes, and mechanisms. *Annals of Behavioral Medicine*.

[11] Ryan P., Maierle D., Mary E. C., Csuka M. E., Thomson A., Szabo A. (2013). Computer-based intervention to enhance self-management of calcium and vitamin D intake in women. *Western Journal of Nursing Research*.

[12] Meiqiu H., Fangyan H. (2012). Effect of health education combined with follow-up on self-management behavior of osteoporotic patients with low back pain. *China Medical Herald*.

[13] Jones C. J., Smith H., Llewellyn C. (2014). Evaluating the effectiveness of health belief model interventions in improving adherence: a systematic review. *Health Psychology Review*.

[14] Xia C., Fang W., Jinmei Z. (2019). Research progress on self-management of chronic diseases. *General Practice Nursing*.

[15] Li H., Liu Y., Li Q., Fan J., Gan L. (2020). Effects of a fast track surgery nursing program in perioperative care of older patients with a hip fracture. *European geriatric medicine*.

[16] Sinclair K. A., Makahi E. K., Shea-Solatorio C., Yoshimura S. R., Townsend C. K. M., Kaholokula J. K.’a. (2013). Outcomes from a diabetes self-management intervention for native Hawaiians and Pacific people: partners in care. *Annals of Behavioral Medicine*.

[17] Ryan P. (2009). Integrated theory of health behavior change. *Clinical Nurse Specialist*.

[18] Dabbo S., Dabbo N. (2010). Motivational interviewing: preparing people for change. *University of Toronto Medical Journal*.

[19] Sanghera S., Frew E., Gupta J. K., Kai J., Roberts T. E. (2017). Sensitivity to scale of willingness‐to‐pay within the context of menorrhagia. *Health Expectations*.

[20] Pang Z., Shan M., Li Y. (2022). The Efficacy of Rehabilitation Nursing Interventions on Patients with Open Lower Limb Fractures. *Journal of Healthcare Engineering*.

[21] Jinxiu W. (2015). Effect of extended nursing intervention on compliance and quality of life of elderly orthopedic patients. *Chinese Contemporary Medicine*.

[22] Li Q., Wang Y., Shen X. (2014). Improvement of Negative Psychological Stress Response in Elderly Patients With Femoral Neck Fracture by Integrated High-Quality Nursing Model of Medical Care. *Frontiers in Surgery*.

[23] Juan Z. (2020). Effect of continuous rehabilitation nursing on rehabilitation exercise compliance, fall risk events and activities of daily living of elderly patients with fracture after discharge. *Nursing Research*.

The article "A Study on the Effect of Nursing Intervention Based on Health Behavior Change Integration Theory on Patients with Limb Fracture and Its Effect on Limb Function and Self-Efficacy" was retracted in 2023. Reasons: signs of a paper mill; suspected computer-generated content; unreliable results or conclusions; lack of ethics approval or compliance.

[24] Kuntz J. L., Safford M. M., Singh J. A. (2014). Patient-centered interventions to improve medication management and adherence: a qualitative review of research findings. *Patient Education and Counseling*.

[25] Lihuan C., Xiaofeng Z. (2018). Effect of targeted nursing based on CGA on functional rehabilitation and postoperative complications of elderly patients with intertrochanteric fracture of femur who underwent PFNA operation. *Nursing Practice and Research*.

[26] Yuhong F., Linyi Z. (2021). Application of sequential rehabilitation nursing program in microrepair of limb fracture with vascular injury. *Chinese Journal of Microsurgery*.

[27] Xueqing D., Zhoulian F., Libing C. (2021). Application of rehabilitation nursing combined with psychological nursing in the treatment of nonunion after limb traumatic fracture with interlocking intramedullary nail. *Qilu Journal of Nursing*.

[28] Wei N., Zhou Y., Chang W., Zhang Y., Chen W. (2017). Displaced intra-articular calcaneal fractures: classification and treatment. *Orthopedics*.

[29] Müller D., Borsi L., Stracke C., Stock S., Stollenwerk B. (2015). Cost-effectiveness of a multifactorial fracture prevention program for elderly people admitted to nursing homes. *The European Journal of Health Economics*.

[30] Sine K., Lee Y., Zullo A. R., Daiello L. A., Zhang T., Berry S. D. (2019). Incidence of lower‐extremity fractures in US nursing homes. *Journal of the American Geriatrics Society*.

[31] Cho H. M., Ha J. S., Seo J. W. (2019). Conservative treatment using a sponge cast for transfer fractures in nursing home patients. *Clinical Interventions in Aging*.

[32] Suyun G., Huiqiong G., Xuejin P. (2016). Study on the effect of health education on secondary fracture of osteoporotic fracture. *Nursing Practice and Research*.

[33] Saito Y., Miura K., Arima H. (2022). Predictors of lower limb fractures in general Japanese: NIPPON DATA90. *Plos one*.

[34] Min Z. (2020). *Application of health education based on ITHBC theory in self-management of middle-aged patients with type 2 diabetes mellitus*.

[35] Fufang C., Feiqin Z., Shuifang W. (2017). The effect of patient management based on health behavior change integration theory on the self-management level of COPD patients. *Chinese Hospital Statistics*.

